RETRACTED

# Effectiveness of GnRH Antagonists and Agonists in Patients with Hormone-Sensitive Prostate Cancer: A Retrospective Study

**DOI:** 10.1155/2022/7608428

**Published:** 2022-06-09

**Authors:** Zhenghao Liu, Chunguang Yang, Xing Zeng, Chunjin Ke, Jihua Tian, Zhihua Wang, Zhiquan Hu

**Affiliations:** Department of Urology, Tongji Hospital of Tongji Medical College, Huazhong University of Science and Technology, Wuhan, China

## Abstract

**Objective:**

To assess the effectiveness of gonadotropin-releasing hormone (GnRH) antagonists and agonists in the treatment of patients with hormone-sensitive prostate cancer (HSPC), thus providing valid data support for their clinical treatment.

**Methods:**

We collected 52 and 65 HSPC patients treated with GnRH antagonists and agonists, respectively, in Tongji Hospital, Tongji Medical College of HUST between May 2019 and April 2021. Prostate-specific antigen (PSA) levels before and after treatment were recorded and analyzed. Further, univariate and multivariate logistic regressions were used to analyze the influencing factors of PSA control rate in HSPC patients.

**Results:**

In patients receiving antagonist, the control rate of prostate-specific antigen (PSA) was 54.28% and 88% without and with abiraterone, respectively, and 47.91% and 72% in patients treated using agonist without and with abiraterone. In 32 pairs of patients obtained via propensity score matching, the PSA control rates were 84.38% and 53.13% for those receiving antagonists and agonists, respectively, and 66.67% and 50% for those without abiraterone, respectively. In addition, univariate logistic regression analysis showed that the type of androgen deprivation therapy (ADT) drugs and combined use of abiraterone had a significant effect on the control rate of PSA. Further multivariate logistic regression revealed that GnRH antagonists in ADT drugs were risk factors for PSA control rate.

**Conclusion:**

The PSA control rate of HSPC patients treated with GnRH antagonist is significantly higher than that of the agonist group, and the use of GnRH antagonist is an independent predictor of PSA control rate.

## 1. Introduction

Prostate cancer (PCa) is the most common nonskin cancer and the second leading cause of cancer-related death in males, with an increasing incidence of approximately 160,000 cases and 366,000 deaths per year [1, 2]. More Chinese prostate cancer patients are diagnosed in the late stage due to low awareness and screening rates [3]. Since the growth of PCa cells is dependent on androgens, androgen deprivation therapy (ADT) is the main treatment for advanced, metastatic, or recurrent PCa [4]. Most patients with metastatic hormone-sensitive prostate cancer (mHSPC) initially respond to ADT [5]. Studies have shown that the 5-year survival rate for metastatic HSPC is only 30% [6]. The purpose of ADT is to inhibit serum testosterone to castration levels, thereby preventing androgen receptor (AR) activation [7]. A significant decrease in prostate-specific antigen (PSA) levels occurs in most patients treated with ADT, and PSA levels may remain low or undetectable for many years, but biochemical recurrences are frequent [8].

RETRACTED

Common drugs for ADT include gonadotropin-releasing hormone (GnRH) agonists and antagonists, which can achieve chemical castration on PCa patients [9, 10]. GnRH agonists act by inhibiting the production of luteinizing hormone (LH) and thus the synthesis of testicular androgens [11]. GnRH antagonists prevent rapid and reversible production of LH and FSH, thereby inhibiting testosterone to depot levels without a flare phenomenon [12]. In order to improve the therapeutic efficacy, GnRH agonists are also combined with antiandrogens as a classic mode for PCa treatment. But even if antiandrogens are used in combination to block adrenal-derived androgens, a significant portion of patients will experience testosterone rebound two weeks after GnRH agonist injection, and present with aggravated symptoms, such as increased bone pain, urinary tract obstruction, and spinal cord compression [13]. And some patients will develop resistance to GnRH agonists [14]. By contrast, degarelix, the new generation of GnRH antagonist, can rapidly inhibit the release of gonadotropins without testosterone rebound and the above clinical symptoms [15, 16]. Previous domestic studies have been limited to GnRH agonists but lack the comparison of the efficacy between antagonists and agonists. Therefore, this study retrospectively collected the clinical data of HSPC patients treated with GnRH antagonists and agonists. Based on collected data, we analyzed and investigated the effectiveness of GnRH antagonists and agonists.

## 2. Materials and Methods

### 2.1. Study Subjects

We collected 52 HSPC patients that received GnRH antagonist therapy and 65 HSPC patients that received GnRH agonist therapy at the Department of Urology, Tongji Hospital, Tongji Medical College of HUST between May 2019 and April 2021. All patients were aged over 18 years. Inclusion criteria were as follows: (1) histologically or cytologically confirmed PCa without ADT; and (2) receiving bone scan, chest and abdomen CT, pelvic MRI, and other examinations before starting treatment to determine TNM staging. Exclusion Criteria were as follows: (1) patients with ADT treatment duration of more than 3 months; (2) patients taking other endocrine drugs except abiraterone and apalutamide during treatment; and (3) patients who were not followed up regularly as required during treatment.

RETRACTED

General data of patients, such as age, TNM stage, Gleason score, and serum PSA baseline concentration, were recorded. Informed consent was obtained from each patient, and this study was approved by the Ethics Committee of Tongji Hospital, Tongji Medical College of HUST (No. TG-IRB20211246).

### 2.2. Treatment Methods

Patients in the antagonist group were subcutaneously injected with degarelix at an initial dose of 240 mg and a maintenance dose of 80 mg, and the injection was given every 28 days. Based on this, 23 patients were treated with 1000 mg abiraterone plus 5 mg prednisone additionally.

Patients in the agonist group were treated with subcutaneous injection of 3.75 mg leuprorelin, subcutaneous injection of 3.6 mg goserelin, or intramuscular injection of 3.75 mg triptorelin. The injection was also given every 28 days. Based on this, 17 patients additionally received 1000 mg abiraterone plus 5 mg prednisone, and the remaining patients were treated with 50 mg oral bicalutamide daily.

### 2.3. Prostate-Specific Antigen (PSA) Test

Fasting blood was collected from patients after receiving ADT in the morning, allowed to stand at room temperature for 2 h, and centrifuged at 3500 × rpm for 10 min. Subsequently, the supernatant was collected and serum PSA levels were measured using an automatic biochemical analyzer (Mindray, China). The time to examine PSA level after receiving ADT treatment was used as the time for the first reexamination, and the postoperative follow-up examination time was 1.5 years. The PSA control rate (>90%) was defined as a PSA decrease of more than 90% from baseline at the time of reexamination.

### 2.4. Statistical Analysis

The experimental results were statistically analyzed using SPSS 26.0. Measurement data with normal distribution were expressed as mean ± standard deviation (SD), and *T* test was used for comparison; measurement data with nonnormal distribution were expressed as median, and Mann–Whitney *U* test was for analysis. Enumeration data was expressed as percentage (%). Propensity score matching (PSM) was adopted, with a module was used for propensity score matching analysis, with a matching tolerance (caliper width) of 0.02 and matching indicators of age, Gleason score, PSA level, TNM stage, and time to first reexamination. Univariate and multivariate logistic regressions were performed to analyze the factors influencing the PSA control rate in HSPC patients. *P* < 0.05 was considered to indicate a statistically significant difference.

## 3. Results

### 3.1. Comparison of the Efficacy between Two Treatments before PSM

In this study, 52 and 65 patients with HSPC treated with GnRH antagonists and agonists, respectively, were included, with no significant differences in average age (67.24 ± 8.873 years *vs*. 68.14 ± 7.557 years), TNM stage (T1-T2: 2 *vs*. 8; T3-T4: 10 *vs*. 13, M1: 40 *vs*. 44), Gleason score (score ≤ 7: 15 *vs*. 18; score > 7: 37 *vs*. 47), and the median time to reexamination (36 days *vs*. 38 days). The PSA control rates were 88% and 62% in patients with abiraterone in the antagonist and agonist groups, respectively, and 54.28% and 47.91% in patients without abiraterone in the two groups. The PSA control rate was higher in the antagonist group than in the agonist group (Table 1).

RETRACTED

### 3.2. Comparison of the Efficacy between Two Treatments after PSM

Since there was a significant difference in PSA levels between the two groups, we then used PSM to increase intergroup comparability. A total of 32 pairs of patients were obtained. After PSM, there was no significant difference between the antagonist group and agonist group in the median time to reexamination (60 days *vs*. 63 days) (Table 2). The PSA control rates of patients with abiraterone were 84.38% and 53.13% in the antagonist group and agonist group, respectively, and 66.67% and 50% in patients without abiraterone in the two groups, respectively. The PSA control rate in the antagonist group was still higher than in the agonist group.

### 3.3. Factors Affecting PSA Control Rate in HSPC Patients after PSM

We next performed univariate and multivariate logistic regression analyses to determine factors influencing PSA control rate in PCa patients after PSM. The univariate analysis results showed that combined use of abiraterone (*P* = 0.011) and GnRH antagonists (*P* = 0.011) was significantly associated with the PSA control rate, suggesting that they might be the influencing factors of PSA control rate for HSPC patients. Multivariate logistic regression analysis of these two factors further showed that GnRH antagonists (*P* = 0.044) had statistical significance, indicating that ADT drugs (antagonists) were independent risk factors in PSA control rate (Table 3).

## 4. Discussion

ADT is the cornerstone for PCa treatment, aiming to rapidly reduce testosterone to castrate levels. The main methods of ADT are surgical castration and medical castration. The drugs used for medical castration are mainly luteinizing hormone-releasing hormone (LHRH) agonists and GnRH antagonists [17]. LHRH acts more slowly, with a high level of testosterone in the first ten days after injection, while GnRH antagonists directly compete with receptors on the pituitary gland and rapidly inhibit the release of gonadotropins without testosterone rebound at the early stage of injection. Moreover, degarelix overcomes the problems of first- and second-generation antagonists, such as short lasting efficacy and the induction of allergic reactions [16, 18, 19], becoming a popular option for medical castration. It has been reported that antagonists can not only achieve the suppression of testosterone secretion through the inhibition of the GnRH receptor, luteinizing hormone secretion and follicle-stimulating hormone secretion, but also significantly reduce the adrenal-derived androgen level in serum [20]. Intermittent treatment with degarelix can maintain the inhibition of PSA and improve sexual function as well as the quality of life [20].

RETRACTED

In this study, we found that the PSA control rate in the antagonist group was significantly higher than that in the agonist group, and the control rate in the antagonist plus abiraterone group was higher than that without abiraterone. The above results were consistent with the study by Matsubara et al. [21]. In order to reduce the evaluation errors, we used PSM to match the baseline data of patients to increase the comparability between the two groups. After PSM, the PSA control rate of patients in the antagonist group was still significantly higher than that of patients in the agonist group. In addition, logistic regression showed that the type of ADT drugs (antagonists) was an independent risk factor for the PSA control rate. A one-year phase III clinical trial by Sun et al. also indicated that the PSA control rate of patients in the two groups by day 364 was 82.3% and 71.7%, respectively (*P* = 0.038); the antagonist group had significantly better effect, suggesting that degarelix was superior to agonist combined with antiandrogens in PSA control during long-term medical castration therapy [22]. In addition, a comprehensive analysis of multiple clinical trials demonstrated that degarelix maintained PSA at better levels compared to GnRH agonists and also improved lower urinary tract symptoms caused by tumors; the antagonist was also superior to agonists in controlling prostate volume and IPSS score [23–25].

This study still has some limitations, such as small sample size (the best sample size is 42 at a type I error rate of 5% and power of 90%), no record of testosterone and PSA levels 3 days after injection, and no data on testosterone during reexamination. The lack of these data limits the analysis accuracy of short-term efficacy of these two groups. This study is designed to explore the advantages of GnRH antagonist, so clinical studies with more than 1 year of follow-up are more conducive to highlighting the advantages. Finally, there are fewer study indicators. Clinical studies have found safety issues with GnRH agonists and antagonists when performing ADT as well, such as cardiovascular disease, metabolic dysfunction, and fractures [26–28]. These all require further larger sample sizes for comparison.

RETRACTED

## 5. Conclusion

In summary, GnRH antagonists have distinct advantages in PSA control over GnRH agonists. A combination of GnRH antagonists and abiraterone may achieve better results in PSA control rates. Collectively, our study provides an effective theoretical basis for the clinical treatment of HSPC.

## Figures and Tables

**Table 1:** Baseline data of the included patients before propensity score matching.

Indicators	Antagonist	Agonist	*P* value
Cases (*n*)	52	65	
Age (year)	67.24 ± 8.873	68.14 ± 7.557	0.547
TNM stage (*n*)			0.225
T1-T2	2	8	
T3-T4	10	13	
M1	40	44	
Gleason score			0.663
≤7 points	15	18	
>7 points	37	47	
PSA control rate (%)			0.001
With abiraterone	88	62	
Without abiraterone	54.28	47.91	
Median time to reexamination (day)	36	38	0.590

**Table 2:** Baseline data of the included patients after propensity score matching.

Indicators	Antagonist	Agonist	*P* value
Cases (*n*)	32	32	
Age (year)	67.03 ± 7.442	66.81 ± 6.301	0.883
TNM stage (*n*)			0.617
T1-T2	2	2	
T3-T4	7	7	
M1	23	23	
Gleason score			0.651
≤7 points	8	9	
>7 points	24	23	
PSA control rate (%)			0.044
With abiraterone	84.38	53.13	
Without abiraterone	66.67	50	
Median value of PSA baseline level (ng/ml)	204.85	211.82	0.864
Median time to reexamination (day)	60	63	0.861

**Table 3:** Univariate and multivariate logistic regression analysis.

Univariate logistic regression analysis				Multivariate logistic regression analysis		
Variables	OR	95% CI	*P* value	OR	95% CI	*P* value
Age	1.017	0.938-1.103	0.684			
TNM stage (M1)	0.769	0.228-2.592	0.672			
Gleason score (≥7)	0.917	0.503-1.670	0.776			
PSA baseline level	2.406	0.717-8.074	0.149			
Reexamination time	1.007	0.995-1.02	0.233			
Combined use of abiraterone	5.079	1.282-20.125	0.011	4.124	0.996-17.079	0.051
ADT drugs (antagonists)	4.375	1.320-14.504	0.011	3.585	1.033-12.435	0.044

## Data Availability

The data used to support the findings of this study are available from the corresponding author upon request.
